The article "miR-146a Inhibited Pancreatic Cancer Cell Proliferation by Targeting SOX7" was retracted in 2023. Reasons: signs of a paper mill; suspected computer-generated content; unreliable results or conclusions; concerns about the data.

# miR-146a Inhibited Pancreatic Cancer Cell Proliferation by Targeting SOX7

**DOI:** 10.1155/2022/2240605

**Published:** 2022-02-16

**Authors:** Chouman Sulidankazha, Wei Han, Tieying He, Hai Lin, Kun Cheng, Xiaohan Nie, Qilong Chen

**Affiliations:** Department of Pancreatic Surgery, Digestive and Vascular Surgery Center, The First Affiliated Hospital of Xinjiang Medical University, Urumqi 830054, Xinjiang Province, China

## Abstract

MicroRNAs (miRNAs) act as a kind of small and noncoding RNA, which have been implicated in the regulation of various pathobiological processes in cancer, including progression in pancreatic cancer and in other human cancers. Previous reports demonstrate that pancreatic cancer has been reported as one of the leading causes of cancer-related death, and some factors including oncogenic genes and environments are involved in tumorigenesis. In our study, we found microRNA-146a (miR-146a) was evidently downregulated in pancreatic cancer tissues and cells. Overexpression of miR-146a obviously reduced cell proliferation and tumorigenesis in vitro, as determined by MTT analysis, colony formation analysis, EdU analysis, and cell cycle experiments. Here, we found tumor suppressor sex-determining region Y-box 7 (SOX7) was the direct target of miR-146a. Overexpression of miR-146a decidedly inhibited SOX7 expression, which promotes cell proliferation and tumorigenesis. Knockdown of miR-146a increased SOX7 expression. Depression of miR-146a and SOX7 promoted cell proliferation and tumorigenesis in vitro, confirming miR-146a regulated pancreatic cancer cell proliferation by inhibiting SOX7. In summary, we found miR-146a reduced the cell proliferation of pancreatic cancer through targeting SOX7. In the present study, we demonstrated the function of miR-146a in pancreatic cancer and might provide a new target in the treatment of pancreatic cancer.

## 1. Introduction

Pancreatic cancer (PC) is defined as a malignancy at digestive tract, featured by insidious initiation and rapid progression [1, 2]. Besides, it has become a significant health problem because it is one of the most frequently diagnosed tumors in humans and the important cause of cancer-related death in humans for a long time [3]. As reported in Global Cancer Statistics 2020, pancreatic cancer remains an important cancer worldwide and is responsible for over 4.5% of the 5.5 million tumor deaths worldwide in 2020, ranking seventh for mortality globally [4]. Accordingly, owing to the lack of effective interventions and the high prevalence, we needed a better understanding of the molecular mechanism of PC development.

MicroRNAs (miRNAs) are small noncoding RNAs which negatively regulate the expression of target genes by binding to the 3′ untranslated regions (UTRs) of the target mRNAs [5]. MicroRNA plays different roles in different cancer types. Given evidence has demonstrated that miRNAs can affect biological behaviors such as proliferation, differentiation, and apoptosis [6]. Previous research studies have proved miR-146a as a specific suppressor miRNA in many kinds of tumors that acts by repressing the expression of the proliferation-associated cancer gene or inhibiting tumor metastasis [7, 8]. However, whether miR-146a influenced pancreatic cancer development has not been reported. Actually, the dbDEMC database showed that miR-146a was obviously downregulated in pancreatic cancer. To further explore whether miR-146a could serve as a promising prognostic marker and to discover their function in PC, we found miR-146a was a tumor suppressor in PC cell lines. Overexpression of miR-146a obviously decreased PC cell line proliferation ability.

Sox genes encode transcription factors that possess strong homology to the high-mobility group (HMG box), which are a family of transcription factors, which have a high-mobility-group DNA-binding domain (HMG box), and they have been reported to play vital roles in embryogenesis [9]. There are at least 30 Sox members expressed in many different cell types and tissues and at multiple stages during development. Sex-determining region Y-box 7 (Sox7), together with Sox17 and Sox18, belongs to the Sox group F subfamily [10]. Sox7 encodes an HMG box transcription factor and has been implicated in parietal endoderm differentiation [11].

A previous study demonstrated that the expression of SOX7 mRNA was frequently downregulated in many human cancer cell lines and tumor tissues [12]. Some members of the SOX family are negative regulators of the WNT-b-catenin-TCF signaling pathway [13]. SOX7, a member of subgroup F along with SOX17 and SOX18, has been reported to regulate hematopoiesis and cardiogenesis originally. Furthermore, accompanied with the increasing evidence, SOX7 in particular has also been revealed to be a tumor suppressor in a number of human cancers [12]. For example, its downregulation was observed in tumors from the ovary, stomach, and lungs [14]. Functionally, studies have proved that overexpression of SOX7 could inhibit hepatocellular carcinoma cell growth, with G1 to S phase arrest. shRNA-mediated SOX7 silencing in nontumorigenic breast cells increased proliferation, migration, and invasion [15]. Conversely, ectopic SOX7 expression inhibits proliferation, migration, and invasion of breast cancer cells in vitro and tumor growth in vivo [16]. Although its role is finely interpreted in multiple human cancers and can be regulated by miRNAs in cancer cells, whether SOX7 can be regulated by miR-146a has not been addressed in pancreatic cancer yet.

Our study confirmed that cancer cell proliferation was regulated positively by SOX7 through miR-146a pancreatic cancer cell proliferation. In the present study, we investigated the role of miR-146a in PC and addressed the mechanism how miR-146a regulates SOX7 in PC. The study might provide a new molecular target for the diagnosis and treatment of PC.

## 2. Materials and Methods

### 2.1. Cell Lines and Cell Culture

Human pancreatic cancer cell lines BxPC3, SW1990, Panc-1, PCI-35, and JF-305 and the normal human pancreatic duct epithelial cell HPC-Y5 were purchased from the American Type Culture Collection (ATCC; Manassas, VA, USA). Cell lines were separately incubated in RPMI 1640 and DMEM (GIBCO, Grand Island, NY, USA) supplemented with 10% fetal bovine serum (Hyclone, Logan, UT, USA) in an atmosphere of 95% air and 5% carbon dioxide at 37°C.

### 2.2. Patients and Tissue Specimens

A total of 52 individuals including 26 patients who were diagnosed with pancreatic cancer (pathologically confirmed as pancreatic cancer) and 26 controls were recruited from the hospital in this study. None of the patients had received any radiotherapy or chemotherapy before sampling. The study was approved by the Ethics Committee of the hospital, and written informed consent was obtained from all participants in advance.

### 2.3. Cell Transfection

The 10^5^ Panc-1 and PCI-35 cells were separately seeded in 6-well plates before transfection. miR-146a was purchased from Gene Pharma (Shanghai, China) for the overexpression of miR-146a. miR-NC was adopted as a control vector. Lentivirus, which could express SOX7 (len-SOX7), was structured by Invitrogen (Carlsbad, CA, USA). The lentivirus empty vector (len-NC) was adopted as the control vector. When cells grew up to approximately 70% of the 6-well plates, Lipofectamine 3000 (Invitrogen, Carlsbad, CA, USA) was used for transfection assays according to the manufacturer's protocol. The transfection process lasted 48 h. For stable cell transfection, cells were selected in culture medium containing 0.4 mg/ml Geneticin (puromycin; Invitrogen). After one month, puromycin-resistant miR-146a upregulation stable cell lines (Panc-1 and PCI-35) were established. RNA interference of SOX7 and NC which were transfected into PCI-35 were designed and synthesized by Gene Pharma Biotech, Shanghai, China. Oligonucleotides used for SOX7 knockdown were as follows: ACGCCGAGCTGTCGGATGG.

### 2.4. Protein Extraction and Western Blot

Transfected cells were lysed with precooled Radio-Immunoprecipitation Assay lysis buffer supplemented with protease inhibitor (Beyotime Institute of Biotechnology, Shanghai, China) for 30 min on ice. The supernatant was collected after centrifugation at 14,000 rpm, 4 °C for 20 min. Protein concentration was determined by a bicinchoninic acid protein concentration determination kit (RTP7102, Real-Time Biotechnology Co., Ltd., Beijing, China). The samples (20 *µ*g) were subjected to 10% sodium dodecyl sulfate-polyacrylamide gel electrophoresis and then transferred to polyvinylidene difluoride membranes (Millipore, Bedford, MA). The blotted membranes were blocked with 3% bovine serum albumin (BSA; Beijing Solebo Biotechnology Co., Ltd, Beijing, China) for 2 h at room temperature, incubated with a primary antibody for 4 °C overnight, washed three times with TBST, and then probed with a secondary antibody for 2 h at room temperature. *β*-Actin was used as a loading control. The levels of the proteins were observed with a chemiluminescence detection system. The primary antibodies were anti-SOX7 (1 : 1 000, R&D System, USA) and *β*-actin (1 : 1000, WeiAo, China). Secondary antibodies were HRP-conjugated goat anti-rabbit antibody (1 : 3000, WeiAo, China) and goat anti-rat antibody (1 : 3000, WeiAo, China).

### 2.5. RNA Extraction

Total RNA extraction from serum samples was performed using TRIzol reagent (Invitrogen, Carlsbad, USA), and the cDNA was synthesized with the First-Strand cDNA Synthesis Kit (Thermo, Waltham, USA) by random priming according to the manufacturer's protocol. The reaction product was quantified by RT-PCR. *β*-Actin was taken as the internal control.

### 2.6. qRT-PCR

For analysis of miR-146a and *β*-actin expression, we employed a two-step qRT-PCR with specific primers. Real-time RT-PCR was performed using a PRISM 7300 Sequence Detection System (Applied Biosystems, CA), in which each reaction (20 ul) contained 10 ul PCR Master Mix (Ambion, TX) and 2.5 ul RT product, and each sample was analyzed in triplicate. PCR was carried out at 95°C for 10 min, followed by 40 cycles of amplification at 95°C for 15 s and 60°C for 60 s. The results are representative of two independent assays. Different cell lines were calculated using the comparative Ct (2 ^–^^△△Ct^) method. The primers used in qPCRs are listed in Table 1.

### 2.7. EdU Assay

The EdU Imaging Detection Kit (KeyGEN BioTECH, China) has been used for the EdU staining assay. In brief, at 48 h posttransfection, the prewarmed EdU staining solution with a final concentration of 10 *μ*M was added to each cell unit and incubated for 2 h at 37°C. The medium was discarded, and the cells were fixed with 4% paraformaldehyde (Sinopharm Chemical Reagent Co., Ltd., China) for 15 min at room temperature. Then the cells were washed two times with PBS containing 3% BSA. 0.5% Triton X-100 (Shanghai Shangbao Biotechnology Co., Ltd, Shanghai, China) in PBS was added to each well and incubated for 20 min at room temperature. The cells were washed two times with PBS containing 3% BSA. The Click-iT reaction solution was added and incubated in the dark at room temperature for 30 min. The cells were stained with Hoechst 33,342 staining solution diluted 1 : 2000 for 15 min and photographed under a laser scanning confocal microscope (LSM780NLO; Zeiss).

### 2.8. Cell Proliferation

Briefly, for cell proliferation, 1,000 cells were seeded in a 96-well plate. Each group was intended with 5 replicate wells. Transfection was performed using the techniques of the cell transfection method. The cells were grown in an incubator and were harvested at different time points (0 h, 24 h, 48 h, 72 h, and 96 h). The CCK-8 (Beyotime, China) of 10 *μ*L was added to the cells in each well and then incubated for 1 h at 37°C. The OD value of each well at 450 nm was measured by a microplate spectrophotometer (ELX-800, BIOTEK, USA).

### 2.9. Flow Cytometry

The PCL-35-control and PCL-35-miR-146a-overexpression cell cycles were determined using the Cell Cycle Detection kit (KeyGEN BioTECH, China). Briefly, the cells were gathered after 48 h of transfection, washed two times with PBS, and centrifuged at 310 g for 5 min. Precooled 70% ethanol was added and fixed overnight at 4°C. The fixed cells were washed twice with PBS, and the supernatant was discarded. A PI/RNase staining solution (RnaseA: PI = 1 : 9) was added and mixed at room temperature for 30–60 min in the dark. Instantly, the cells were analyzed via a flow cytometer (NovoCyte, ACEA Biosciences, Inc., USA).

### 2.10. Dual Luciferase Reporter Assay

The wild-type and mutant SOX7 30 untranslated region (3′UTR) sequences were amplified by polymerase chain reaction and ligated into the pMIRREPORT luciferase vector (Ambion, Austin, TX, USA) to yield pMIR-SOX7 30-UTR (SOX7 30-UTR). The HEK293 cells were seeded into the six-well plates and allowed to reach 60–80% confluence. The cells were then cotransfected with wild-type/mutant SOX7 30-UTR and miR-9mimic/miR-NC using Lipofectamine 2000. 24 hours later, the cells were harvested and lysed. Luciferase reporter assay was performed on the Dual-Luciferase Reporter Assay System (Promega, Madison, WI, USA) according to the manufacturer's instructions. The firefly luciferase activity was normalized to Renilla luciferase activity.

Luciferase assays were carried out as described below. Briefly, cells were cotransfected with luciferase reporter constructs, miRNA and Renilla using Lipofectamine^TM^ 2000 (Invitrogen), and Firefly and Renilla luciferase activities were measured after 48 h with a Dual-Luciferase_Reporter Assay System (Promega) using a luminometer.

The wild-type (wt) sequences of SOX7 that contain binding sites with miR-146a or mutant type (mut) sequences that do not contain them were synthetized. The former sequences were then inserted into the pmirGLO vector (Promega, Madison, WI, USA). The miR-146a-overexpression or control was cotransfected with the vectors into PCL-35 cells, and the luciferase activities were detected using the Dual-Luciferase Reporter Assay System (Promega, Madison, WI, USA). We used Renilla luciferase activity as a normalized control.

### 2.11. Statistical Analysis

All statistical analyses were conducted using GraphPad Prism 8 (GraphPad) for Mac OS. Experiments were repeated 3 times unless otherwise stated, and the representative results were shown. Quantitative data are expressed as mean ± SEM. A two-tailed *t*-test was used to identify significant differences in comparisons unless otherwise stated. For all statistical analyses, the level of significance was set at 0.05.

## 3. Result

### 3.1. miR-146a Was Downregulated in Pancreatic Cancer

First off, we found miR-146a was obviously downregulated in pancreatic cancer tissues compared with tumor adjacent tissues (Figure 1(a)).  Figure 1(b) shows that miR-146a expression in five different pancreatic cancer cells, such as BxPC3, SW1990, Panc-1, PCL-35, and JF-305l, was compared with normal human pancreatic duct epithelial cell HPC-Y5 by qRT-PCR assays. We found miR-146a was downregulated in pancreatic cancer cells in RNA expression. Moreover, we found overexpression of miR-146a in PC caused a better prognostic effect months after operation by clinical result (Figure 1(c).

### 3.2. miR-146a Suppressed the Proliferation of Pancreatic Cancer Cells

Although we had known miR-146a was downregulated in pancreatic cancer, to confirm the function of miR-146a in pancreatic cancer cell lines, we established lentiviral-mediated stable overexpression of miR-146a in Panc-1 and PCL-35 cells (Figures 2(a) and 2(b)). We found overexpression of miR-146a evidently inhibited and suppressed the proliferation of pancreatic cancer cells. Initially, the effects of miR-145 on the proliferation of Panc-1 and PCL-35 cells were investigated using a CCK-8 assay (Figures 2(c) and 2(d)). Besides, Figures 2(e) and 2(f) show overexpression of miR-146a suppressed the proliferation of Panc-1 and PCL-35 cells by EdU assays. In order to explore the role of miR-146a in the cell cycle, we found overexpression of miR-146a arrested the Panc-1 and PCL-35 cells at S phase (Figure 2(g)). Taken together, miR-146a overexpression inhibited pancreatic cancer cell proliferation and tumorigenesis in vitro.

### 3.3. SOX7 Is a Direct Target of miR-146a in Pancreatic Cancer Cells

Previous research had confirmed that overexpression of miR-146a inhibited pancreatic cancer cell proliferation. In order to explore the mechanism, we searched for the target gene of miR-146a. It was predicted that SOX7 might be a potential direct molecular of miR-146a by the bioinformatics online analysis software, TargetScan 7.2 database (http://www.targetscan.org/vert_71/) (Figure 3(a)). We then synthesized wt or mut SOX7 luciferase vectors according to the binding site between 3′-UTR region of SOX7 and miR-146a. Luciferase reporter assays showed that the activities could be reduced by miR-146a in wt groups but not in mut groups or miR-NC groups (Figure 3(b)). Moreover, qRT-PCR found that the miR-146a mRNA level could be noticeably decreased by miR-146a (Figures 3(c) and 3(d)). Besides, western blot analysis showed that overexpression of miR-146a could decrease the SOX7 protein level (Figures 3(e) and 3(f)). Accordingly, these data demonstrated that SOX7 was a target of miR-146a, which was negatively regulated by miR-146a in Panc-1 and PCL-35 cells.

### 3.4. miR-146a Inhibited Pancreatic Cancer Cell Proliferation by Downregulating SOX7

We found that cell proliferation marker protein Ki67 expression was significantly reduced and apoptosis marker protein BAX expression increased when miR-146a was upregulated in PCL-35 by western blot (Figure 4(a)). Furthermore, we found that cell Ki67 protein expression was significantly reduced and BAX protein expression increased when SOX7 was upregulated in PCL-35 by western blot (Figure 4(b)). In order to confirm that miR-146a depressed cell proliferation and tumorigenesis in vitro by inhibiting SOX7, we overexpressed SOX7 in PCL-35 cells with miR-146a overexpression.  Figure 4(c) shows that overexpression of miR-146a inhibited Ki47 protein expression and inhibited cell proliferation in PCL-35 which was increased by overexpression of SOX7. Moreover, the effects of miR-146a could be reversed by SOX7 upregulation (Figure 4(c)). Taken together, SOX7 was the target gene of miR-146a in pancreatic cancer cells. miR-146a inhibited cell proliferation and tumorigenesis in vitro by inhibiting SOX7.

## 4. Discussion

In the present study, we observed the downregulation of miR-146a in the human pancreatic cancer cell lines tested (BxPC3, SW1990, Panc-1, PCI-35, and JF-305) compared with the normal human pancreatic duct epithelial cell HPC-Y5, as well as in pancreatic tumor tissues by clinical results. We also discovered that overexpression of miR-146a in pancreatic cancer cells depressed pancreatic cancer cell proliferation and arrested the Panc-1 and PCL-35 cells at S phase by flow cytometry assays. Consequently, we concluded that overexpression of miR-146a reduced pancreatic cancer cell proliferation and might be a potential therapeutic target in pancreatic cancer.

Previously, research indicated that miR-146a played an important role of anti-oncogene through downregulating the expression levels of multiple oncogenes in tumor [17]. Induction of miR-146a by multiple myeloma cells in mesenchymal stromal cells stimulates their protumoral activity. Furthermore, the miR-146a gene was reported to downregulate NF-*κ*B, suppress cell proliferation, and induce apoptosis, and therefore might function as a potent tumor suppressor [18]. The miR-146a-5p/TRAF6/NF-kB p65 axis regulates pancreatic cancer chemoresistance [19]. Upregulation of miR-146a contributes to the inhibition of the invasion of pancreatic cancer cells. Our research found that miR-146a inhibited pancreatic cancer progression.

It has been well established that SOX7 influences many kinds of cancer progression. In a recent study, Guo et al. demonstrated that the SOX7 gene was downregulated in 47% of the pancreatic adenocarcinomas, and tumor-specific inactivation of SOX7 by promoter hypermethylation was found in 48% of the primary pancreatic tumors tested [20]. These authors also suggested that SOX7 serves as an independent checkpoint for b-catenin function in pancreatic and colon epithelial cells [21, 22]. Furthermore, many research studies indicated that SOX7 could be regulated to influence cancer progression or apoptosis by miRNAs [23]. Knockdown of miR-935 increases paclitaxel sensitivity via regulation of SOX7 in non-small-cell lung cancer. miR-935 promotes gastric cancer cell proliferation by targeting SOX7, and miR-935 promotes liver cancer cell proliferation and migration by targeting SOX7 [24, 25].

In the present study, an important molecular association between miR-146a and SOX7 was demonstrated. Firstly, the bioinformatics analysis indicated that SOX7 may be one of the potential targets for miR-146a. Subsequently, it was identified that miR-146a is markedly downregulated in PC tissues, which is consistent with a previous study. More importantly, a significant negative correlation was observed between miR-146a and SOX7 expression in PC tissues, and the expression of SOX7 was decreased in PCL-35 cells accompanied by suppressed cell proliferation when overexpressing miR-146a, suggesting that miR-146a may be involved in the regulation of SOX7 in PC. This hypothesis was further supported by the luciferase activity assay, in which the data demonstrated that miR-146a was able to directly target the 3′UTR of SOX7 and the binding site was consistent with the seed region predicted by TargetScan. These data demonstrated that miR-146a may inhibit cell proliferation of PCs by targeting SOX7.

In conclusion, we established in this study the role of miR-146a in PC and its target gene SOX7. We also clarified the mechanisms that miR-146a targeted SOX7 in pancreatic cancer. miR-146a could induce pancreatic cancer cell apoptosis and inhibit cell proliferation, and this may be achieved through suppressing SOX7 expression. The data presented in this report represent the attempt to disclose the role of miR-146a in suppressing pancreatic cancer, which may be useful in the development of new therapeutic strategies for pancreatic cancer.

## Figures and Tables

**Figure 1:** miR-146a was downregulated in pancreatic cancer. (a) miR-146a was observably downregulated in pancreatic cancer tissues compared with tumor adjacent tissues. (b) miR-146a was observably downregulated in five pancreatic cancer cells compared with normal human pancreatic duct epithelial cell HPC-Y5 by qRT-PCR. (c) Survival relevance analysis of miR-146a expression in pancreatic cancer. According to the qRT-PCR data, the expression of miR-146a was classified into low expression (*n* = 26) and high expression (*n* = 26) (^*∗*^*P* < 0.05; ^*∗∗*^*P* < 0.01; ^*∗∗∗*^*P* < 0.001).

**Figure 2:** miR-146a suppressed the proliferation of pancreatic cancer cells. (a, b) Viability in Panc-1 and PCL-35 cells transfected with control or miR-146a. (c, d) CCK8 analysis of Panc-1 and PCL-35 cells transfected with control or miR-146a. (e, f) miR-146a inhibited the proliferation ability in pancreatic cancer cells Panc-1 and PCL-35, as determined by 5-ethynyl-2′-deoxyuridine (EDU) incorporation assays (scale bar, 25 *µ*m; magnification, ×400). (g) The cell cycle distribution of miR-146a inhibited the proliferation ability in pancreatic cancer cells. PCL-35 cells infected with miR-146a lentivirus or control vector were analyzed as described in Materials and Methods (^*∗*^*P* < 0.05; ^*∗∗*^*P* < 0.01; ^*∗∗∗*^*P* < 0.001).

**Figure 3:** SOX7 is a direct target of miR-146a in pancreatic cancer cells. (a) Predicted interacting sites between miR-146a and SOX7 were showed including wilt type and mutant type. (b) Luciferase reporter activities of wild-type SOX7 vectors were decreased by miR-146a but not miR-NC or mutant SOX7 vectors in PC cells. (c, d) miR-146a inhibits SOX7 RNA expression in Panc-1 and PCL-35 by qRT-PCR. (e, f) miR-146a inhibits SOX7 protein expression in Panc-1 and PCL-35 by western blot (^*∗*^*P* < 0.05; ^*∗∗*^*P* < 0.01; ^*∗∗∗*^*P* < 0.001).

**Figure 4:** miR-146a inhibited pancreatic cancer cell proliferation by downregulating SOX7. (a) Overexpression of miR-146a decreased Ki67 protein expression and increased BAX protein expression in PCL-35 by western blot. (b) Overexpression of SOX7 increased Ki67 protein expression and decreased BAX protein expression in PCL-35 by western blot. (c) Overexpression of SOX7 promoted Ki67 protein expression and inhibited BAX protein expression in PCL-35 cells which were, respectively, inhibited and promoted by overexpression of miR-146a through western blot (^*∗*^*P* < 0.05; ^*∗∗*^*P* < 0.01; ^*∗∗∗*^*P* < 0.001).

**Table 1:** The sequences of primers for RT-PCR in this study.

Gene name	Sequences (5′–3′)
miR-146a: forward	CGCGTGAGAACTGAATTCCA
miR-146a: reverse	AGTGCAGGGTCCGAGGTATT
SOX7: forward	GCCAAGGACGAGAGGAAAC
SOX7: reverse	GTTGGGGTAGTCCTGCATGT
*β*-Actin: forward	CTACGTCGCCCTGGACTTCGAGC
*β*-Actin: reverse	GATGGAGCCGCCGATCCACACGG

## Data Availability

The data used to support the findings of this study are available on reasonable request from the corresponding author.
